# Efficacy and Safety of Apatinib plus Neoadjuvant Chemotherapy for Locally Advanced Esophageal Squamous Cancer: A Phase II Trial

**DOI:** 10.1155/2022/4727407

**Published:** 2022-07-18

**Authors:** Bo Yang, Xiaofeng Guo, Cheng Le, Wenzhong Su, Xiaoming Li, Yanfeng Zhang, Guangyi Yang, Weimin Liang, Zhixin Zheng, Junpeng Wu, Yaowen Zhang, Anlin Hao

**Affiliations:** Department of Thoracic Oncology, Anyang Tumor Hospital, The Affiliated Anyang Tumor Hospital of Henan University of Science and Technology, Henan Medical Key Laboratory of Precise Prevention and Treatment of Esophageal Cancer, Anyang, 455000, China

## Abstract

Evidence for neoadjuvant chemotherapy combined with targeted therapy for locally advanced esophageal squamous cancer (ESCC) is inadequate. We conducted a single-arm phase II trial to evaluate the efficacy and safety of apatinib combined with taxol and cisplatin (ATP) for locally advanced ESCC. All patients were cT3-4aN0-3 M0 (IIIb-IVa) stage, which were confirmed by histopathology. Apatinib was taken orally (425 mg/d) for two cycles, followed by one cycle of rest. Taxol was administered at 135 mg/m^2^ intravenously on day 1, and cisplatin was administered at 20 mg/m^2^ intravenously on day 1 to day 3. Radical ESCC resection was performed 4 weeks after ATP. The primary endpoint was pathological response rate (pCR). Secondary endpoints were pathologic response rate (MPR), disease-free survival (DFS), overall survival (OS), R0 resection rate, and safety profile. This trial was registered. We evaluated 41 patients for screening from Oct 2018 to July 2020, of whom 39 were enrolled in the study, with a median age of 65 years (range 49-75 years), and 29 (74.4%) were male. Among the 39 patients, 1 was considered unresectable by the multidisciplinary team due to tumor progression, and 38 patients underwent surgery eventually. The median follow-up was 22 months (range 5-29 months), and the follow-up rate was 100%. The 1-year and 2-year OS was 95% and 95%, and the 1-year and 2-year DFS was 85% and 82%, respectively. Thirty-eight (97.3%) successfully underwent R0 resection. Of the 38 evaluable patients, 9 (23.6%) were pCR, and 15 (39.5%) were MPR. The most common ATP-related AEs were nausea (76.9%), leucopenia (53.8%), neutropenia (51.2%) and vomit (51.2%), anemia (41.0%), and hypertension (25.6%). The most frequent grade 3-4 events included leucopenia (15.3%), neutropenia (15.3%), nausea (12.8%), vomit (12.8%), and hypertension (10.2%). No treatment-related death occurred. Neoadjuvant apatinib combined with taxol and cisplatin for locally advanced ESCC showed favorable activity and manageable safety.

## 1. Introduction

Esophageal cancer (EC) is the tenth most common malignancy in terms of incidence and the sixth leading cause of cancer-related death worldwide, and locally advanced EC accounts for nearly half of cases [1]. Esophageal squamous cell carcinoma (ESCC) accounts for more than 90% of the Asian population, and more than half of the global ESCC cases occur in China [2]. Surgery plays an important role in the treatment of EC. However, most patients undergoing radical resection have a high rate of recurrence and metastasis and a poor prognosis [3]. Indeed, the 5-year overall survival (OS) for all EC patients is 15%-25%, compared with less than 4% for patients with metastatic disease [4]. This has led to a shift in management strategies from monotherapy to multimodality regimens. Neoadjuvant therapy has been tested to reduce locoregional and distant recurrence and improve survival [5, 6].

In the field of neoadjuvant therapy, based on the results of CROSS study [7] and NEOCRTEC5010 [8], neoadjuvant chemoradiotherapy (nCRT) has become the standard treatment for locally advanced esophageal carcinoma which can be resected surgically and is recommended by the guidelines. In fact, in the clinical practice of resectable local advanced esophageal cancer in China, surgeons were concerned about perioperative complications, nCRT accounted for less than 5%, and more neoadjuvant chemotherapy was used. After neoadjuvant therapy, patients who reached pCR had a longer survival time [7, 8]. For neoadjuvant chemotherapy, the pCR rate of patients in previous studies was less than 10% [9]. In order to achieve a significant increase in pCR rates and improve the survival benefit of patients, it is imperative to explore a new protocol.

Antiangiogenic therapy may be a better add-on option than conventional chemotherapeutic agents [10]. Antiangiogenic agents include antivascular endothelial growth factor (VEGF) antibodies and VEGF receptor (VEGFR) tyrosine kinase inhibitors (TKIs). Mesylate apatinib, a small molecule oral tyrosine kinase inhibitor (TKI) that mainly targets VEGF2, had shown definite antitumor activity and controllable side effects in many human cancers [11, 12]. A previous phase II study showed that apatinib was effective as second- or further-line treatment for advanced EC [13]. Given the current evidence on apatinib for ESCC, we designed a trial to evaluate the efficacy and safety of apatinib combined with taxol and cisplatin (ATP) as neoadjuvant therapy for locally advanced ESCC in China.

## 2. Methods

### 2.1. Study Design and Patients

This was a single-arm, open-label, phase II trial conducted in our hospital between October 2018 and July 2020. Inclusion criteria included age at 18-75 years, histologically proven, previously untreated, clinical diagnosis of locally advanced ESCC, cT3-4aN0-3 M0 (IIIb-IVa) evaluated by computed tomography (CT) and laparoscopy, Eastern Cooperative Oncology Group (ECOG) performance status (PS) of 0-1, and adequate organ function. Patients with at least one measurable lesion (according to Response Evaluation Criteria in Solid Tumours [RECIST], version 1.1 [14]) were eligible. Patients with pregnant and lactating women, tumor bleeding, esophageal perforation, and esophageal fistula were excluded, and history of prior or concurrent malignancies, known allergies to apatinib or any of the study drugs, a definite gastrointestinal bleeding tendency and/or coagulation disorders (international normalized ratio > 1.5), uncontrolled blood pressure, and prior myocardial infarction within 6 months were excluded from the study. This study was approved by the Ethics Committee of Anyang Tumor Hospital. All patients received written informed consent before enrollment. This study was registered in the China Trial Register (http://ChiCTR.gov.cn), with the identification number ChiCTR19000221783.

### 2.2. Preoperative ATP Treatment and Assessment

ATP regimen consisted of apatinib 425 mg/day continuously, intravenous taxol 135 mg/m^2^ on day 1, and cisplatin 20 mg/m^2^ intravenously on day 1 to day 3. This regimen was repeated every 3 weeks until unacceptable toxicity, up to 2 cycles. Four weeks after completing two cycles of ATP, enhanced CT of the neck, chest, and upper abdomen and/or positron emission tomography CT (PET-CT) and ultrasound endoscopy was carried out. Tumor response was assessed by two senior radiologists according to NCI-proposed Response Evaluation Criteria in Solid Tumors, version 1.1 (RECIST 1.1) [14, 15]. Adverse events (AEs) were graded according to the National Cancer Institute Common Terminology Criteria for Adverse Events (NCI-CTCAE 4.0). The assessed clinical response included complete response (CR), partial response (PR), stable disease (SD), and progressive disease (PD). Dosage adjustments including interruptions and reductions were allowed for the management of treatment-related adverse events (AEs).

### 2.3. Surgery and Assessments

Surgery was scheduled 28-42 days after the second treatment cycle. Surgical indication was based on the efficacy of ATP treatment to determine the possibility of radical resection. A multidisciplinary team consisting of experienced radiologists, oncologists, and surgeons confirmed that whether the patient was eligible for surgery. All resected specimens were examined by the same pathologist to assess the extent of residual disease, stage of disease, and efficacy of preoperative treatment. Pathological response rate (pCR) was defined as no viable tumor cells in resected tumor specimens, and major pathologic response (MPR) was defined as ≤10%. The primary end point was pCR rate. Secondary endpoints were MPR rate, disease-free survival (DFS), overall survival (OS), margin-free (R0) resection rate, downstaging, and safety profile. Pathologic response was evaluated and graded using post-ATP resection materials, according to the Classification of Esophageal Carcinoma, 8^th^ edition [16]. The definition of complications was based on the International Consensus on Standardization of Data Collection for Complications Associated With Esophagectomy [17].The severity of postoperative complications was assessed according to the Clavien-Dindo classification of surgical complications. The first follow-up was 1 month after surgery. Follow-up was performed every 3 months for 2 years and every 6 months for 2-5 years until the end of the trial or death.

### 2.4. Statistical Analysis

Demographic data, outcome data, and other clinical parameters were presented as the frequency for categorical variables and the median with interquartile range (IQR) for age variable. Statistical analysis was undertaken using SPSS 26.0 (IBM Corp). A 2-sided *p* value <0.05 was considered to be statistically significant.

## 3. Results

### 3.1. Patient Characteristics

From October, 2018 to July 1, 2020, 41 eligible patients were enrolled after signing informed consent documents. The study flow diagram was shown in Figure 1. 1 patient experienced unacceptable toxicity, and 1 patient withdrew from the study. And 39 patients were evaluated for tumor response. Baseline characteristics of all 41 patients were listed in Table 1. There were 29 males and 10 females, with a median age of 65 years (49-75 years). Tumors were located in upper esophagus in 8 cases (20.5%), middle in 30 cases (76.9%), and lower in 1 case (2.6%), respectively. At baseline, 36(92.4%) patients had AJCC Eighth Edition-defined stage IIIb disease, while the other 3(7.6%) patients were defined as stage IVa disease. All treated patients had an ECOG PS of 0 (74.4%) or 1 (25.6%). All patients underwent surgery after two-cycle neoadjuvant therapy and received two-cycle adjuvant chemotherapy.

### 3.2. Neoadjuvant Treatment and Toxicity

33 patients received full-dose chemotherapy, while 6 patients required dose reductions, including 4 with a dose reduction in taxol and 2 in both cisplatin and taxol. Treatment administration was delayed in 2 patients due to neutropenia (*n* = 1) and thrombocytopenia (*n* = 1). During neoadjuvant ATP therapy, all 39 patients had any grade AEs, and 10 (34.5%) patients experienced AEs of grades 3 or 4. The ATP-related AEs are listed in Table 2. The most common ATP-related AEs were nausea (76.9%), leucopenia (53.8%), neutropenia (51.2%) and vomit (51.2%), anemia (41.0%), and hypertension (25.6%). The most common treatment-related > grade III AEs included leucopenia (15.3%), neutropenia (15.3%), nausea (12.8%), vomit (12.8%), and hypertension (10.2%). No treatment-related death occurred.

### 3.3. Surgical Treatment and Complication

Among 39 patients, 1 case was considered unresectable by the multidisciplinary team due to tumor progression, and 38 patients underwent surgery eventually. Minimally invasive esophagectomy (McKeown) and open esophagectomy were received by 36 (94.8%) and 2 (5.2%) patients, respectively. The median duration from the last administration of apatinib to surgery was 35.5 ± 2.5 days. Among 38 patients, 37 underwent R0 resection, and 1 underwent R1 resection (for positive resection margins). R0 resection rate was 97.3% (37/38). Because of tumor adhesion and azygos vein arch, two patients suffered blood loss 1700 ml and 1100 ml, respectively, during surgery. The average bleeding amount in operation was 264.4 ± 23.7 ml. Anastomotic leakage rate was 10.5%, wound infection rate was 7.8%, and pulmonary infection rate was 18.4%. The median hospitalization was 18.6 ± 2.3 days. There were no perioperative deaths, reoperation, intensive care unit admissions, or readmission.

### 3.4. Radiological and Pathological Response

According to the RECIST 1.1 criteria, 39 patients who received neoadjuvant ATP therapy achieved objective response: 17 (43.6%) achieved CR, 16 (41.0%) achieved PR, 5 (12.3%) achieved SD, and one had progressive disease (PD). The ORR and DCR were 84.6% and 97.2%, respectively (Figures 2 and 3, Table 3). Of the 38 evaluable patients who underwent surgery, 9 (23.6%) were pCR, 15 (39.5%) were MPR, and 19 (48.7%) achieved downstaging after surgery (Table 4). No significant association was identified pathological response and smoking status, drinking status, clinical TNM stage, and primary tumor location.

### 3.5. Overall Survival

All patients were followed up until May 10, 2021. The follow-up time was 5-31 months (median: 22 months), and the follow-up rate was 100%. The 1-year and 2-year OS of the 38 patients was 95% and 95%, and the DFS was 85% and 82%, respectively (Figure 4).

## 4. Discussion

nCRT is the standard treatment for locally advanced ESCC and can provide long-term survival benefits compared to surgery alone [7]. In the real world, the implementation rate of nCRT in China was not high, which might be related to China's national conditions and the late development of ESCC multidisciplinary therapy. Based on the results of clinical studies such as OEO2 [18] and JCOG9907 [19], preoperative treatment of EC in China was still dominated by chemotherapy. Although neoadjuvant chemotherapy had been recommended for resectable ESCC patients, the 5-year overall survival rate was poor. Therefore, apatinib combined with taxol and cisplatin was used in this study to explore its efficacy and safety.

Antiangiogenic therapy was associated with potentially serious toxic effects, such as gastrointestinal perforation, hemorrhage, and delayed wound-healing, presenting additional challenges to neoadjuvant chemotherapy. Previous clinical trials had shown that patients with several solid tumors receive apatinib at dose of 500-850 mg/day [20]. Considering the toxicity of TP, we used 425 mg/day as the initial dose of apatinib in this study. Apatinib was given for 2 continuous cycles, and surgery was scheduled 4 weeks after the end of neoadjuvant ATP therapy.

Regarding safety, all patients completed neoadjuvant TPA therapy. The incidence of grade 3-4 AEs was 34.5%. All AEs during ATP therapy were tolerated and controllable, suggesting that preoperative addition of apatinib to TP chemotherapy was safe. No treatment-related death occurred. The incidence of surgery-related complications was 36.8%, among which anastomotic leakage (10.5%), wound infection (7.8%), and pulmonary infection (18.4%) were the most common complications. Only 2 cases suffered blood loss for tumor adhesion and azygos vein arch hemorrhage during surgery. Fortunately, no patient underwent reoperation, and no intensive care unit stay or readmission occurred. The interval between ATP and surgery induced the negative impact of ATP regimen on surgery.

Complete surgical resection (R0 resection) was an important predictor of long-term survival in EC [21]. In this study, among the 38 patients, 37 underwent R0 resection, the R0 resection rate was 97.3%, and one underwent R1 resection (for positive surgical margins). pCR was proved to be associated with long-term survival [7, 8]. Of the 38 evaluable patients, 9 (23.6%) were pCR, and 15 (39.5%) were MPR. The commendable downstaging of overall TNM stage was noted (48.7%). The 1-year and 2-year OS was 95% and 95%, and the 1-year and 2-year DFS was 85% and 82%, respectively. In this study, we selected patients with cT3-4aN0-3 M0 (IIIb-IVa) stage at a relatively late stage, efficacy results showed that ESCC patients responded well to neoadjuvant ATP and surgery, and their tumors shrank. We expected that ATP regimen will bring higher pCR rate and more survival benefits and also provide a certain prospect for waiting and observing nonsurgical treatment strategies in the treatment of locally advanced ESCC. With the development of multiomics technology and medical science and technology, accurate screening, accurate evaluation, and multidisciplinary comprehensive treatment will surely make great progress, and it will no longer be far away for patients with locally advanced ESCC to retain esophageal function, high quality of life, and long-term survival.

Our trial had some limitations. First, this was a single-arm trial, without control group or randomization; so, selection bias could not be ruled out. Second, the number of cases was small, and the follow-up time was short; so, it was still necessary to expand the sample size and increase follow-up time.

In conclusion, neoadjuvant apatinib plus paclitaxel and cisplatin had manageable treatment-related toxicity. This regimen induced relatively high pCR, demonstrating its antitumor efficacy in locally advanced ESCC.

## Figures and Tables

**Figure 1:** Flow diagram.

**Figure 2:** Waterfall plots for clinical tumor response.

**Figure 3:** CT images of a case who reached pCR pre-TPA and post-TPA treatment ((a) for esophageal tumor of pre-TPA, (b) for esophageal tumor of post-TPA, (c) for positive lymph node of pre-TPA, and (d) for positive lymph node of post-TPA).

**Figure 4:** Kaplan-Meier plot of 38 ESCC patients ((a) for OS and (b) for DFS).

**Table 1:** Baseline characteristics.

Variable	Patients (*N* = 39)
Sex, *N* (%)	
Male	29 (74.4)
Female	10 (25.6)
Age (years), *N* (%)	
>60	27 (69.3)
≤60	12 (30.7)
ECOG performance status, *N* (%)	
0	29 (74.4)
1	10 (25.6)
Primary tumor location, *N* (%)	
Upper	8 (20.5)
Middle	30 (76.9)
Lower	1 (2.6)
cT stage	
T3	26
T4a	13
cN stage	
N1	21
N2	16
N3	2
cTNM stage, *N* (%)	
IIIb	36 (92.4)
IVa	3 (7.6)
Hypertension, *N* (%)	
Yes	7 (17.9)
No	32 (82.1)
Smoking, *N* (%)	
Yes	10 (25.6)
No	29 (74.7)
Drinking, *N* (%)	
Yes	22 (56.4)
No	17 (43.6)

**Table 2:** Incidence of adverse events during neoadjuvant treatment.

Adverse events	Any grade, *n* (%)	Grades 3/4, *n* (%)
Hematological		
Leukopenia	21 (53.8)	6 (15.3)
Neutropenia	20 (51.2)	6 (15.3)
Anemia	16 (41.0)	2 (5.1)
Thrombocytopenia	5 (12.8)	1 (2.5)
Nonhematological		
Hypertension	10 (25.6)	4 (10.2)
Proteinuria	3 (7.6)	1 (2.5)
Hand-foot syndrome	1 (2.5)	0 (%)
Aminotransferase increased	2 (5.1)	1 (2.5)
Hyperbilirubinemia	1 (2.5)	0 (0)
Naupathia	30 (76.9)	5 (12.8)
Vomiting	20 (51.2)	5 (12.8)
Stomachache	1 (2.5)	0 (0)

**Table 3:** Primary assessment method: overall assessment.

Parameter	N/(%)
Number of patients screened	41
Number of patients enrolled	39
Number of patients completed two cycles of neoadjuvant therapy	39
Number of patients evaluated toxicity	39
Number of patients evaluated tumor response	39
Number of patients received surgery	38
Radiological response	RECIST 1.1
CR	17 (43.6%)
PR	16 (41.0%)
SD	5 (12.3%)
PD	1 (2.5%)
ORR	84.6%
DCR	97.2%
R0 resection	37 (97.3%)
Pathological response	
pCR	(93.6%)
MPR	15 (39.5%)
Downstaging rate	19 (48.7%)
Lymph nodes involved	
ypN0	20 (51.35)
ypN1	11 (28.2%)
ypN2	6 (15.4%)
ypN3	2 (5.1%)

**Table 4:** Surgical-related complications.

Parameter	*N* (%)
Surgical method	
VATS McKeown radical esophagectomy under thoracoscope	36 (94.8%)
Radical resection of esophageal carcinoma with three incisions on the right side	1 (2.6%)
Esophageal carcinoma with two incisions on the left chest and neck	1 (2.6%)
Anastomotic leakage	4 (10.5%)
Wound infection rate	3 (7.8%)
Pulmonary infection rate	7 (18.4%)
The average bleeding amount in operation	264.40 ± 23.7 ml
The median hospitalization	18.6 ± 2.3 days

## Data Availability

All the underlying data supporting the results of our study are in the manuscript.
